RETRACTED

# Lifestyle Improvements and Vitamin D Supplementation Play an Important Role in the Prevention of Childhood Diabetes

**DOI:** 10.1155/2022/6133908

**Published:** 2022-10-04

**Authors:** Erdi Xu, Chunyan Yin, Xiaoqing Yi, Yuesheng Liu

**Affiliations:** Department of Pediatric, The Second Affiliated Hospital of Xi'an Jiaotong University, Xi'an, Shaanxi, China

## Abstract

**Objective:**

This study was to investigate the characteristics of insulin secretion and the 25-hydroxyvitamin D3 (25(OH)D3) levels in children with obesity.

**Methods:**

A retrospective analysis was conducted among children who underwent health checkups in the pediatric healthcare department of our hospital from January 2018 to January 2021, and they were divided into a normal group and an obese group according to their BMI. The insulin secretion and the 25(OH)D3 levels of the two groups of children were compared. A total of 721 children were included in the study, including 591 in the normal group and 130 in the obese group, with an obesity rate of 18.03%.

**Results:**

The blood glucose of the normal group was 4.55 ± 1.75 mmol/L, and the 2 h PG was 7.51 ± 2.11 mmol/L; in the obesity group, they were 6.03 ± 2.16 mmol/L and 8.92 ± 3.24 mmol/L, respectively. The FPG and 2 h PG in the obese group were significantly higher than those in the normal group (all *P* < 0.05). The incidence of IFG/IGT in the normal group was 5.24% (31/591), and the incidence of DM was 3.71% (22/591); the incidence of IFG/IGT in the obese group was 14.62% (19/130), and the incidence of DM was 13.08% (17/130). The incidences of IFG/IGT and DM in the obese group were significantly higher than those in the normal group (*P* < 0.05). The FINS of the children in the normal group was 18.46 ± 3.15 *μ*U/mL, and the HOMA-IR was 2.64 ± 0.62; the above indicators in the obese group were 19.11 ± 4.72 *μ*U/mL and 3.01 ± 0.83, respectively. The FINS and HOMA-IR in the obese group were significantly higher than those in the normal group (*P* < 0.05). The serum 25(OH)D3 level in the normal group was 28.15 ± 5.27 ng/mL, of which 556 cases were normal in 25(OH)D3 and 35 cases were deficient in 25(OH)D3. The serum 25(OH)D3 level in the obese group was 24.35 ± 4.51 ng/mL, of which 112 cases were normal in 25(OH)D3 and 18 cases were deficient in 25(OH)D3. The level of serum 25(OH)D3 in the normal group was significantly higher than that in the normal group, and the ratio of 25(OH)D3 deficiency was significantly lower than that in the normal group (*P* < 0.05).

**Conclusions:**

The blood glucose level of childhood obesity was significantly increased, the incidence of abnormal glucose metabolism and diabetes was significantly increased, and the level of 25(OH) vitamin D3 was significantly decreased. Lifestyle improvements and vitamin D supplementation play an important role in the prevention of childhood diabetes. Because the major causes of childhood obesity are excessive caloric intake and lack of exercise, the most effective and direct measures to prevent obesity are a reasonable lifestyle, reasonable eating habits, and moderate exercise. Although genetics are critical, there is no reliable way to eliminate obesity genes in the human body. Therefore, the role of obesity genes is required to be ultimately eliminated by reduced caloric intake and increased physical activity.

RETRACTED

## 1. Introduction

In recent years, with the advances of people's living standards, the probability of children being diagnosed with obesity has increased year by year. Childhood obesity is a disease that endangers health. Unlike pathological obesity caused by abnormal metabolism, it is a morbid feature caused by excess nutrition in children. It threatens children's physical and mental health and quality of life, as well as children's ability to socialize. Childhood obesity is a major global public health problem, and the growing prevalence of childhood obesity has led to the emergence of multiple serious obesity-related comorbidities, threatening children's health and placing enormous pressure on healthcare [1, 2]. In addition, childhood obesity persists into adulthood, especially in severely obese children [3]. Early-onset type 2 diabetes has been linked to progressive neuropathy, retinopathy to blindness, nephropathy to chronic renal failure, and atherosclerotic cardiovascular disease to significant consequences such as stroke, myocardial infarction, and sudden death, as evidenced by previous studies [4]. Obesity, a condition of excess fat, is always measured using body mass index (BMI) due to the nonavailability of the direct measurement of body fat and high cost. Children with a BMI of more than 22 kg/m^2^ are considered obese [5]. In addition, obesity in children can easily lead to other chronic diseases, such as hypertension, heart disease, and diabetes, constituting considerable morbidity and mortality of chronic diseases in children in adulthood.

Immune-mediated type 1 diabetes is predominant in children and adolescents, but the incidence of type 2 diabetes caused by obesity has also increased dramatically in recent years. It has been confirmed that obesity is closely related to insulin resistance, together with the lack of insulin, resulting in type 2 diabetes [6, 7]. Serum 25(OH)D is the most abundant metabolite in circulation and can be used as an indicator for assessing systemic vitamin D status. Vitamin D deficiency is highly prevalent among children worldwide, and mild deficiency of vitamin D is common even in healthy children [8]. Statistics from the United States, Norway, and China show that children with serum 25(OH)D < 50 nmol/L are considered vitamin D deficient [5]. Vitamin D plays an important role in maintaining immune function and can prevent infection, autoimmune diseases, tumors, and type 2 diabetes [9–11]. A prospective finding also suggests that vitamin D supplementation in infants and early childhood reduces the incidence of type 1 diabetes.

RETRACTED

In type 2 diabetes, the main pathological changes are impaired pancreatic *β* cell function, insulin resistance, and systemic inflammatory response. Studies have shown that vitamin D3 is involved in the progression of type 2 diabetes. Vitamin D3 may play a role in pancreatic *β* cells by mediating the binding of circulating 25-hydroxyvitamin D3 (25(OH)D3) to the pancreatic *β* cell vitamin D receptor [12]. In addition, vitamin D can also activate 25(OH)D3 through 1-alpha hydroxylase expressed in *β* cells [13]. To further confirm the relationship between childhood obesity, insulin metabolism characteristics, and 25(OH)D3, this study specifically investigates children with obesity and healthy children admitted to the Children's Health Department of our hospital.

## 2. Materials and Methods

### 2.1. Study Design

A retrospective analysis was conducted among children who underwent health checkups in the pediatric healthcare department of our hospital from January 2018 to January 2021, and they were divided into a normal group and an obese group according to their BMI. A total of 721 children were included in the study, including 591 in the normal group and 130 in the obese group, with an obesity rate of 18.03%.

The randomization was carried out using an online web-based randomization tool (freely available at http://www.randomizer.org/). For concealment of allocation, the randomization procedure and assignment were managed by an independent research assistant who was not involved in screening or evaluation of the participants.

For sample size calculation, the sample size was determined according to the hospital sampling survey case-control study method, the estimated prevalence was 5%, the relative error of the sampling survey was 20% and set at 1.5, with a 95% confidence interval, Za = 1.96 and a 10% data incompleteness rate, and the final calculated sample size was in the range of 35 to 50.

If the parameter beta is either a difference of means, a log odds ratio or a log hazard ratio, then it is reasonable to assume that *b* is unbiased and normally distributed.

The study protocol and all amendments were approved by the appropriate ethics committee at each center. The study was done in accordance with the protocol, its amendments, and standards of clinical practice. All participants provided written informed consent before enrolment, Ethics No. HU-YU20180102.

RETRACTED

The basic data, insulin metabolism characteristics, and 25(OH)D3 level were compared. A total of 721 children were included in the study, including 591 in the normal group and 130 in the obese group, with an obesity rate of 18.03%. As shown in Table 1, there was no significant difference in the basic data of the two groups of children and they were comparable.

### 2.2. Inclusion and Exclusion Criteria

Inclusion criteria: (1) aged 0-12 years; (2) the obese group met the BMI cutoff for obesity in children and adolescents aged 0-18, and the BMI of the normal group was within the normal range; and (3) the medical records were complete.

Exclusion criteria: (1) pathological obesity caused by hypothyroidism, hypercortisolism, genetic metabolic disease, and kidney disease; (2) application of drugs that affect blood sugar; (3) anorexia nervosa, eating disorders, etc.; and (4) mental illness.

### 2.3. Observation Indicators

(1) Blood sugar examination: fasting insulin level (FINS), fasting blood glucose (FPG), and 2-hour postprandial blood glucose (2 h PG) were measured by oral glucose tolerance test, and impaired fasting glucose (IFG) and impaired glucose tolerance (IGT) were calculated. (2) Insulin homeostasis: the homeostasis model assessment of insulin resistance (HOMA‐IR) = (FPG × FINS/22.5) was used to evaluate insulin homeostasis. (3) 25(OH)D3 level: fasting peripheral blood was collected from children, and enzyme-linked immunosorbent assay (ELISA) was used to determine the level of 25(OH)D3.

### 2.4. Statistical Methods

The normality of the sample was determined with the Shapiro–Wilk test. Descriptive statistical data were evaluated with the exploratory analyses of the Tukey test. Quantitative mean data (PES/WES, ISQ, and B.L.) were assessed with the nonparametric Wilcoxon-Mann–Whitney *U* test to analyze the inferential statistical.

SPSS 22.0 software was used to organize and statistically analyze the data. The mean ± standard deviation (±*s*) and rate (%) were used to represent measurement data and count data, respectively, and *t*-test and chi-square test were used to compare the differences between groups. The difference was considered statistically significant at *P* < 0.05.

## 3. Results

### 3.1. Blood Sugar Levels

The blood glucose of the normal group was 4.55 ± 1.75 mmol/L, and the 2 h PG was 7.51 ± 2.11 mmol/L; in the obesity group, they were 6.03 ± 2.16 mmol/L and 8.92 ± 3.24 mmol/L, respectively. The FPG and 2 h PG in the obese group were significantly higher than those in the normal group (*P* < 0.05, Table 2).

RETRACTED

### 3.2. Incidence of IFG/IGT and DM

The incidence of IFG/IGT in the normal group was 5.24% (31/591), and the incidence of DM was 3.71% (22/591); the incidence of IFG/IGT in the obese group was 14.62% (19/130), and the incidence of DM was 13.08% (17/130). The incidences of IFG/IGT and DM in the obese group were significantly higher than those in the normal group (*P* < 0.05, Table 3).

### 3.3. FINS and HOMA-IR

The FINS of the children in the normal group was 18.46 ± 3.15 *μ*U/mL, and the HOMA-IR was 2.64 ± 0.62; the above indicators in the obese group were 19.11 ± 4.72 *μ*U/mL and 3.01 ± 0.83, respectively. The FINS and HOMA-IR in the obese group were significantly higher than those in the normal group (*P* < 0.05, Table 4).

### 3.4. 25(OH)D3 Levels

The serum 25(OH)D3 level in the normal group was 28.15 ± 5.27 ng/mL, of which 556 cases were normal in 25(OH)D3 and 35 cases were deficient in 25(OH)D3. The serum 25(OH)D3 level in the obese group was 24.35 ± 4.51 ng/mL, of which 112 cases were normal in 25(OH)D3 and 18 cases were deficient in 25(OH)D3. The level of serum 25(OH)D3 in the normal group was significantly higher than that in the normal group, and the ratio of 25(OH)D3 deficiency was significantly lower than that in the normal group (*P* < 0.05, Table 5).

## 4. Discussion

With the advancement of social living standards and changes in dietary structure, the incidence of childhood obesity is increasing. Childhood obesity immensely hinders the function of various organs, intelligence, and growth and development of children, but also may lead to adult obesity and seriously damage the physical and mental health of children. Additionally, some studies have shown that there is a link between childhood obesity and the onset of chronic diseases such as hyperlipidemia, diabetes, and hypertension in adulthood. Therefore, it is vital to control the weight of children with childhood obesity. Childhood obesity shows propensity towards groups within 1 year old, 5 to 6 years old, or adolescents and is closely related to fast eating and irregular eating [14]. Long-term childhood obesity can lead to various childhood and adult diseases such as hyperlipidemia, hypertension, coronary heart disease, fatty liver, and diabetes [15]. Type 2 diabetes is the result of multiple factors, including genetic, physiological, and lifestyle-related obesity, among which obesity is an important factor in type 2 diabetes [8]. In recent years, the incidence of type 2 diabetes in children has increased significantly and is closely related to childhood obesity.

RETRACTED

In this study, a total of 721 children were included, of which 130 were obese children, and the incidence of obesity was 18.03%. This study confirmed that the FPG and 2 h PG in the obese group were significantly higher than those in the normal group, the incidence of IFG/IGT and DM in the obese group were significantly higher than those in the normal group, and the FINS and HOMA-IR in the obese group were significantly higher than those in the normal group. As is known, FPG and 2 h PG are the main methods for evaluating and diagnosing diabetes, and HOMA-IR is an index used to evaluate the level of insulin resistance in individuals. With the increase of insulin resistance level, the HOMA-IR index will be higher than 1, and these results confirm that blood glucose metabolism is insufficient in children with obesity. Obese children are susceptible to insulin resistance, which reduces insulin sensitivity and increases blood sugar and leads to diabetes [9, 10]. Insulin dysfunction in diabetes can also cause abnormal lipid metabolism, further aggravating dyslipidemia in obese children. Studies have shown that up to 25% of obese children are associated with type 2 diabetes, which is consistent with the results of this study [11].

In this study, the serum 25(OH)D3 level in the normal group was significantly higher than that in the normal group, and the ratio of 25(OH)D3 deficiency was significantly lower than that in the normal group. To our best understanding, 25(OH)D3 is the main form of vitamin D in the body, which can regulate blood calcium levels and affect cell differentiation. The role of vitamin D in the pathophysiology of type 2 diabetes remains controversial [16]. There is increasing evidence that vitamin D plays an important role in reducing the risk of developing diabetes, and vitamin D plays an important role in pancreatic *β* cell dysfunction, impaired insulin action, and systemic inflammation in type 2 diabetes [17]. In an observational study of 6000 subjects examining the relationship between vitamin D levels and the prevalence of type 2 diabetes, there was a significant inverse association between vitamin D levels and diabetes incidence [18].

Studies have shown that in vitamin D-deficient type 2 diabetic patients, vitamin D supplementation not only improves glucose metabolism but also reduces the dosage of oral hypoglycemic agents and insulin [19]. The relationship between vitamin D and diabetes may be related to inhibiting the activity of nuclear factor *κ*B and inflammatory response, increasing the insulin sensitivity pathway and inhibiting the insulin resistance pathway, and accelerating glucose metabolism [20]. The possible explanations are as follows. (1) Cognitive misunderstanding: most parents consider that the fat baby is not associated with lack of nutrition, so the obese child cannot secure vitamin D supplementation. (2) Insufficient absorbable vitamin D and calcium: most of the obese children included in this paper were artificially fed within 1 year of age. (3) The obese children generally grow faster than children of their peer and need more vitamin D. (4) The fat metabolism of the obese children interrupts the metabolism of vitamin D. In recent years, studies have shown that there is a negative correlation between vitamin D and obesity [21]. After a 10% weight loss, a low-calorie diet increased 25(OH)D levels, and this increase was primarily associated with improvements in insulin resistance. (5) Vitamin D is essential for the body to make leptin. Lipoleptin is a hormone that controls food intake and makes people feel full and stop eating [22]. When vitamin D deficiency leads to a decrease in lipid leptin in the body, thus stimulating appetite and causing obesity. In addition, recent studies suggest that VD inhibits the occurrence of obesity by regulating calcium metabolism in vivo, inhibiting parathyroid hormone secretion, and avoiding cellular calcium influx [23].

RETRACTED

Childhood obesity is a nutritional disorder in which energy intake exceeds human consumption for a long time, excess fat accumulation, and weight exceeds a certain range. With the change of dietary structure, the improvement of people's living standards, and the change of lifestyle, childhood obesity is increasing, which blocks children's growth and development, psychology, physique, intelligence, and behavior and seriously affects children's quality of life [24, 25]. Childhood obesity is also a contributor in the increased morbidity and mortality of many chronic noncommunicable diseases in adulthood, making it an increasingly serious global public health problem [26]. The results of this study suggest that lifestyle improvements and vitamin D supplementation play an important role in the prevention of childhood diabetes. It also provides a certain theoretical value for future clinical diagnosis and treatment and direction for drug design against vitamin D.

The participants in this trial are from inpatients in the pediatric department of our hospital, which is relatively single; the sample size is small, and the observation period is not long enough, so the clinical results have certain bias; the supplementation of vitamin D and the improvement of lifestyle in the subject have not been adjusted for different individuals, which leads to deficiencies; this study is a clinical study, and there is no animal experiment, so it lacks a more scientific basis. Future studies, therefore, are required to expand the sample size from multiple centers and observation period and add outcome indices that reflect the coordination of drugs and life, such as more indicators of safety, to obtain more reliable data and provide promising implications.

RETRACTED

In conclusion, the blood glucose level of childhood obesity was significantly increased, the incidence of abnormal glucose metabolism and diabetes was significantly increased, and the level of 25(OH) vitamin D3 was significantly decreased. Lifestyle improvements and vitamin D supplementation play an important role in the prevention of childhood diabetes.

## Figures and Tables

**Table 1:** Baseline data.

	Normal group (*n* = 591)	Obese group (*n* = 130)	*t*/*χ*^2^	*P*
Gender (male/female)	382/209	77/53	1.346	0.246
*Age*				
Mean age (*x* ± *s*, year)	13.45 ± 5.46	12.68 ± 5.29	1.464	0.144
0~3	84	24	1.635	0.651
4~6	195	42		
7~9	116	25		
10~12	196	39		

**Table 2:** Blood glucose levels in two groups of children ($\bar{x}\pm \text{s}$, mmol/L).

	FPG	2 h PG
Normal group (*n* = 591)	4.55 ± 1.75	7.51 ± 2.11
Obese group (*n* = 130)	6.03 ± 2.16	8.92 ± 3.24
*t*	8.347	6.186
*P*	<0.001	<0.001

**Table 3:** Comparison of the incidence of IFG/IGT and DM ($\bar{x}\pm \text{s}$, mmol/L).

	IFG/IGT	DM
Normal group (*n* = 591)	31	22
Obese group (*n* = 130)	19	17
*χ* ^2^	14.50	18.22
*P*	<0.001	<0.001

**Table 4:** Comparison of fasting insulin levels and insulin resistance index.

	FINS ($\bar{x}\pm \text{s}$, *μ*U/mL)	HOMA-IR ($\bar{x}\pm \text{s}$)
Normal group (*n* = 591)	18.46 ± 3.15	1.34 ± 0.32
Obese group (*n* = 130)	19.11 ± 4.72	1.67 ± 0.43
*t*	5.04	9.95
*P*	<0.001	<0.001

**Table 5:** Comparison of 25(OH)D3 levels.

	25(OH)D3	Normal 25(OH)D3	25(OH)D3 deficiency
Normal group (*n* = 591)	28.15 ± 5.27	556	35
Obese group (*n* = 130)	24.35 ± 4.51	112	18
*t*/*χ*^2^	7.629	9.824	
*P*	<0.001	<0.001	

## Data Availability

All data generated or analyzed during this study are included in this published article.
